The article "Metformin inhibits the proliferation of benign prostatic epithelial cells" was retracted in 2024. Reasons: errors in the data; errors in the methods; errors in the images; errors in the text.

# Metformin inhibits the proliferation of benign prostatic epithelial cells

**DOI:** 10.1371/journal.pone.0173335

**Published:** 2017-03-02

**Authors:** Zongwei Wang, Xingyuan Xiao, Rongbin Ge, Jijun Li, Cameron W. Johnson, Cyrus Rassoulian, Aria F. Olumi

**Affiliations:** 1 Department of Urology, Massachusetts General Hospital, Harvard Medical School, Boston, Massachusetts, United States of America; 2 Department of Urology, Wuhan Union Hospital, Huazhong University of Science and Technology, Wuhan, China; 3 Department of Pathology, University of Massachusetts Medical School, Worcester, Massachusetts, United States of America; 4 Shanghai Children 's Medical Center, Shanghai Jiaotong University School of Medicine, Shanghai, China; Medizinische Universitat Innsbruck, AUSTRIA

## Abstract

**Objective:**

Benign prostatic hyperplasia (BPH) is the most common proliferative abnormality of the prostate affecting elderly men throughout the world. Epidemiologic studies have shown that diabetes significantly increases the risk of developing BPH, although whether anti-diabetic medications preventing the development of BPH remains to be defined. We have previously found that stromally expressed insulin-like growth factor 1 (IGF-1) promotes benign prostatic epithelial cell proliferation through paracrine mechanisms. Here, we seek to understand if metformin, a first line medication for the treatment of type 2 diabetes, inhibits the proliferation of benign prostatic epithelial cells through reducing the expression of IGF-1 receptor (IGF-1R) and regulating cell cycle.

**Methods:**

BPE cell lines BPH-1 and P69, murine fibroblasts3T3 and primary human prostatic fibroblasts were cultured and tested in this study. Cell proliferation and the cell cycle were analyzed by MTS assay and flow cytometry, respectively. The expression of IGF-1R was determined by western-blot and immunocytochemistry. The level of IGF-1 secretion in culture medium was measured by ELISA.

**Results:**

Metformin (0.5-10mM, 6-48h) significantly inhibited the proliferation of BPH-1 and P69 cells in a dose-dependent and time-dependent manner. Treatment with metformin for 24 hours lowered the G_2_/M cell population by 43.24% in P69 cells and 24.22% in BPH-1 cells. On the other hand, IGF-1 (100ng/mL, 24h) stimulated the cell proliferation (increased by 28.81% in P69 cells and 20.95% in BPH-1 cells) and significantly enhanced the expression of IGF-1R in benign prostatic epithelial cells. Metformin (5mM) abrogated the proliferation of benign prostatic epithelial cells induced by IGF-1. In 3T3 cells, the secretion of IGF-1 was significantly inhibited by metformin from 574.31pg/ml to 197.61pg/ml. The conditioned media of 3T3 cells and human prostatic fibroblasts promoted the proliferation of epithelial cells and the expression of IGF-1R in epithelial cells. Metformin abrogated the proliferation of benign prostatic epithelial cells promoted by 3T3 conditioned medium.

The article "Metformin inhibits the proliferation of benign prostatic epithelial cells" was retracted in 2024. Reasons: errors in the data; errors in the methods; errors in the images; errors in the text.

**Conclusions:**

Our study demonstrates that metformin inhibits the proliferation of benign prostatic epithelial cells by suppressing the expression of IGF-1R and IGF-1 secretion in stromal cells. Metformin lowers the G2/M cell population and simultaneously increases the G0/G1 population. Findings here might have significant clinical implications in management of BPH patients treated with metformin.

## Introduction

BPH is the most common, proliferative abnormality of the human prostate affecting elderly men throughout the world. Half of all men, ages 51–60, have histologically identifiable BPH and by age 85, the prevalence increases to approximately 90% [1]. In the setting when medical therapy becomes ineffective, prostatectomy by open surgery or transurethral resection of the prostate is considered the primary method of treatment [2]. However, these surgical treatments are often associated with multiple complications, e.g. urinary tract infection, strictures, sexual dysfunction, and blood loss. Meanwhile, the underlying molecular alterations that can potentially be used for targeted therapies are still poorly understood. Further comprehension of the pathophysiology of BPH and development of a more effective approach would be beneficial to the management of BPH.

Accumulation of epidemiologic evidence demonstrates that BPH is associated with diabetes mellitus, i.e, diabetes increases the risk of BPH [3]. In 1966, one of the first publications reported that diabetes was more frequently diagnosed among the patients who subjected to prostatectomy than those who were not [4]. More recently, in a series of early cross-sectional studies, Hammarsten’s group reported a direct correlation between insulin levels and annual BPH growth rates in diabetic patients [5–7]. Other groups further confirmed that hyperinsulinemia and insulin resistance are independent risk factors in BPH development [8, 9]. Together, these studies suggested that BPH is directly associated with diabetes.

Our previous study investigated the molecular mechanism for the development of BPH and demonstrated that IGF-1 plays a critical role during BPH progression [10]. IGF-1 shares many similar sequences with insulin, and performs a fundamental role in the regulation of a variety of cellular processes such as proliferation, differentiation, apoptosis, extracellular matrix expression, chemotaxis, and neovascularization [11–13]. We have found that IGF-1 regulates the stromal-epithelial interaction through the paracrine pathway, and also that the activation of IGF-1R promotes the proliferation of prostatic epithelial cells via MAPK/AKT/cyclin D pathway [10].

The article "Metformin inhibits the proliferation of benign prostatic epithelial cells" was retracted in 2024. Reasons: errors in the data; errors in the methods; errors in the images; errors in the text.

Metformin is a first line medication for type 2 diabetes treatment and has been prescribed to almost 120 million people worldwide [14]. Interestingly, recent studies have suggested this medication as a potential anti-proliferative agent. In prostatic cancer cell lines, metformin has been demonstrated to inhibit cell proliferation and block the cell cycle in the G_0_/G_1_ stage by activating the AMPK pathway [15, 16]. However, the effect of metformin on benign prostatic cells still remains unclear. Here, we show that metformin inhibits the proliferation of two benign prostatic epithelial cell lines, BPH-1 and P69, in a dose-dependent and time-dependent manner. We show that the administration of metformin lowers the G2/M cell population in both cell lines and abrogated the effect of IGF-1 on cell proliferation. Finally, we demonstrate that both the secretion of IGF-1 in fibroblasts and prostatic epithelial cell proliferation promoted by a conditioned medium (CM) of fibroblasts are inhibited by metformin. Our findings suggest that beyond the treatment of diabetes, metformin can also inhibit the proliferation of prostate epithelial cells, which may be beneficial to the treatment of BPH.

## Materials and methods

### Cell culture

Immortalized human benign prostatic epithelial cells, BPH-1 and P69, mouse embryonic fibroblast 3T3 cells were kindly provided by Drs. Simon Hayward (Vanderbilt University, Nashville, TN) and Timothy C. Chambers (University of Arkansas for Medical Sciences, Little Rock, AR), respectively. The cells were maintained in RPMI 1640 (Thermo Scientific, Waltham, MA, USA; for BPH-1and P69) or Dulbecco’s modified Eagle’s medium (DMEM, Thermo Scientific, Waltham, MA, USA; for 3T3) and supplemented with 2 mmol/L glutamine, 10% fetal bovine serum (FBS), and 1% penicillin-streptomycin at 37°C with 5% CO_2_. Human primary prostatic fibroblast cells were the gift of Dr. Douglas Strand (UT Southwestern Medical Center, Dallas, TX). Cells were cultured in Stromal Cell Medium SCGM Bullet Kit^™^ (Lonza, CC-3204 & CC-4181, Walkersville, MD). Conditioned medium (CM) from fibroblast cells were harvested after 24 hours of culture with or without 5 mM metformin. BPH-1 and P69 cells were cultured in CM for 24 hours.

### Reagents

Antibodies to GAPDH, IGF-1, IGF-1R, pho-IGF-1R, pho-IRS-1(Ser636/639), extracellular signal-regulated kinase (ERK), pho-ERK(Thr202/Tyr204), pho-AKT (Ser473), AKT, PARP, cyclin D1, cyclin D2, cyclin D3 and horseradish peroxidase-conjugated secondary antibodies (goat anti-mouse and goat anti-rabbit) were purchased from Abcam (Cambridge, MA, USA), Millipore (Billerica, MA, USA), and Cell Signaling (Danvers, MA, USA). Recombinant mouse IGF-1, anti-human IGF-1 and anti-mouse IGF-1 enzyme-linked immunosorbent assay (ELISA) kit were obtained from R&D Systems (Minneapolis, MN, USA). MTS (3-(4,5-dimethylthiazol-2-yl)-5-(3-carboxymethoxyphenyl)-2-(4-sulfophenyl)-2H-tetrazolium) was from Promega (Madison, WI, USA).

The article "Metformin inhibits the proliferation of benign prostatic epithelial cells" was retracted in 2024. Reasons: errors in the data; errors in the methods; errors in the images; errors in the text.

### Cell proliferation assays

Cell proliferation was measured using the MTS assay and Ki-67 immunostaining. The MTS method was performed in accordance with the manufacturer’s instructions. In brief, MTS substrates were added and incubated for 1 hour at 37°C. Absorbance was measured at 490 nm by a microtiter plate reader. Viability of untreated cells was set to 100%, and the absorbance of wells with only the medium was set to zero. Each experiment was repeated three times. The nuclear protein Ki-67, an indicator of cell proliferation [17] was used as another marker to detect cell proliferation by immunofluorescence staining.

### Immunostaining

As described previously [18], cells grown on glass coverslips were fixed in 4% paraformaldehyde, permeabilized with 0.2% Triton X-100/PBS, and stained with antibodies. The sections were counterstained with DAPI and mounted with mounting medium (Vector Lab, Burlingame, CA, USA).

### Cell cycle assays

We used flow cytometry (BD FACSAria I cell sorter) to assess the population of cells in each phase. Briefly, cells were trypsinized, washed twice in ice-cold PBS, resuspended in staining solution (100μg/ml Ribonuclease inhibitor, 100μg/ml propidium iodide solution, 0.1% NP40 in PBS), and finally incubated for 30 minutes in the dark at RT, prior to analysis.

### Protein extraction and western-blot

The complete cell lysates were harvested on ice with M-PER protein extraction reagent (Thermo Scientific, Waltham, MA, USA) containing a mixture of protease and phosphate inhibitors (Thermo Scientific, Waltham, MA, USA). After sonication for 10 seconds, cell debris was removed by centrifugation (12,000g) for 10 minutes at 4°C. The protein concentration was determined by BCA protein assay reagent (Pierce, Rockford, IL, USA). A total of 50ng of protein per lane was supplemented with loading buffer (NuPage; Invitrogen, Carlsbad, CA, USA) and boiled for 10 minutes. Immunoblotting was performed as previously described [18]. The cell lysates were subjected to 8%-16% Bis-Tris gels (Invitrogen, Carlsbad, CA, USA) and transferred onto PVDF membranes (Millipore, Billerica, MA, USA). Membranes were probed with target antibodies.

The article "Metformin inhibits the proliferation of benign prostatic epithelial cells" was retracted in 2024. Reasons: errors in the data; errors in the methods; errors in the images; errors in the text.

### ELISA

An ELISA kit for IGF-1 was purchased from R&D Systems Inc. (catalog no. MG100), and was used throughout the experiments. The assays were performed in accordance with the instructions of the manufacturer. After completion of the ELISA assay, luminescence was assayed by a plate reader at 450 nm.

### Statistical analyses

The experimental results were presented as mean ± standard error of the mean of replicate analysis accompanied by the number of independent experiments. Statistical analyses were performed using the student’s t-test. A p value of less than 0.05 was considered statistically significant.

## Results

### Metformin inhibits the proliferation of BPH epithelial cells

To investigate the effects of metformin on the proliferation of benign prostate cells, P69 and BPH-1 cells were first maintained in serum-starved conditions for 12 hours. This was followed by the administration of metformin at a concentration of 0.5, 1, 5, or 10 mM. After 24 hours of exposure, a significantly decreased cell viability was observed with escalating doses of metformin (BPH-1, Fig 1A and P69, Fig 1B). Next, P69 and BPH-1 cells were treated with metformin (5 mM) over a 48 hour period. The MTS test showed that metformin inhibited the proliferation of both cell lines in a time-dependent manner (Fig 1C and 1D). The treatment of metformin at 5 mM for 48 hours significantly inhibited the cell growth in both cell lines (p<0.001).

**Fig 1:** Metformin inhibits human benign prostatic epithelial cell growth. A-B: Cell viability of BPH-1 (A) and P69 (B) 24 hours after treatment with various doses of metformin. MTS test was performed as described in Materials and Methods. The results are expressed as percent of viable cells compared with control group. C-D: Cell viability of BPH-1 (C) and P69 (D) after the treatment of 5 mM metformin in different times. *, *P*<0.05; **, *P*<0.001 compared with control group.

### Metformin inhibits IGF-1-induced cell growth of BPH-1 and P69

Since it has been well established that locally enforced IGF-1 expression induces hyperplasia in the prostate [19] [14], we next sought to determine whether metformin regulates cell growth when promoted by IGF-1. As expected, pre-treatment of IGF-1 (100 ng/mL) for 24 hours significantly stimulated the proliferation of BPH-1 (Fig 2A) and P69 cells (Fig 2B). Furthermore, the administration of metformin completely abrogated IGF-1 (100 ng/mL) induced growth in BPH-1(Fig 2A, 2C and 2E) and P69 cells (Fig 2B, 2D and 2F). To further confirm this finding, we evaluated the expression of the proliferative marker, Ki-67, in BPH-1 and P69 cells [17]. We found that metformin markedly decreased the number of Ki-67 positive cells in the BPH-1 (Fig 2C and 2E) and P69 cell lines (Fig 2D and 2F) either with or without IGF-1 treatment. Findings here suggest that metformin inhibits the proliferation of benign prostate epithelial cells, and this effect may be associated with the IGF-1 axis.

The article "Metformin inhibits the proliferation of benign prostatic epithelial cells" was retracted in 2024. Reasons: errors in the data; errors in the methods; errors in the images; errors in the text.

**Fig 2:** Metformin inhibits IGF-1-induced growth of BPH-1 and P69 cells. A-B: Cell viability (MTS test) of BPH-1 (A) and P69 (B) 24 hours after treatment of 100 ng/mL IGF-1 with/without 5 mM metformin. C-D: Representative picture of Ki-67 staining in BPH-1 (C) and P69 (D) cells 24 hours after treatment of 100 ng/mL IGF-1 with/without 5 mM metformin. E-F: Quantification of Ki-67 staining in BPH-1 (E) and P69 (F). *, *P*<0.05 compared with the control group; #, *P*<0.05 compared with the IGF-1 group. CTR: non-treated control, Met: metformin.

### Metformin inhibits the expression of IGF-1R and abrogates IGF-1-induced phosphorylation of IGF-1R

Previously we have shown that IGF-1 signaling plays a critical role in the progression of BPH and also that cyclin D is the main target of IGF-1 signaling pathway [10]. Others have demonstrated the effect of metformin on cell growth is cyclin D-dependent but not mediated by AMPK [15]. We next asked the question if metformin could regulate the activation of IGF-1R. We found that the protein level of pho-IGF-1R was significantly decreased in BPH-1 cells upon the treatment of metformin in a time- and dose-dependent manner (Fig 3A). Metformin also inhibited the phosphorylation of IRS-1, which is one of the primary substrates of IGF-1R (Fig 3A). The ratios of pho-IGF-1R to IGF-1R and pho-IRS-1 to GAPDH were decreased 30 to 100-fold in metformin-treated BPH-1 cells when compared with the untreated control cells (Fig 3B and 3C). Similar results were obtained in P69 cells (data not shown). Furthermore, we observed that metformin not only inhibited the original expression of pho-IGF-1R on BPH-1 (Fig 3D upper panel and Fig 3F) and P69 cells (Fig 3E upper panel and Fig 3G), but also significantly inhibited the IGF-1-stimulated pho-IGF-1R expression (Fig 3D lower panel and Fig 3E lower panel). Together, we speculate that metformin inhibits prostate epithelial cell growth via preventing the IGF-1R expression through autocrine or paracrine mechanisms.

**Fig 3:** Metformin inhibits expression of IGF-1 receptor (IGF-1R) and abrogates IGF-1-induced phosphorylation of IGF-1R. A: Immunoblotting of IGF-1R, pho-IGF-1R and pho-IRS-1 in proliferating BPH-1 cells treated with various doses of metformin for 24 hours, or with 5 mM metformin for the indicated times. B-C: Quantification of the immunoblot protein expression of pho-IGF-1R (B) and pho-IRS-1 (C) in BPH-1 cells treated with 5 mM Metformin for 24 hours, and normalized to IGF-1R or GAPDH, respectively. **, *P*<0.001 compared with control group. D-E: Representative immunofluorescence images of pho-IGF-1R in BPH-1 (D) and P69 (E) cells after exposure to 100 ng/mL IGF-1 in the presence or absence of 5 mM metformin for 48 hours. F-G: Immunoblotting of pho-IGF-1R and pho-IRS-1 in BPH-1 (F) and P69 (G) cells 48 hours after treatment of IGF-1(100 ng/mL) and metformin (5 mM). CTR: untreated control, Met: metformin.

The article "Metformin inhibits the proliferation of benign prostatic epithelial cells" was retracted in 2024. Reasons: errors in the data; errors in the methods; errors in the images; errors in the text.

### Metformin inhibits the expression of cell proliferating regulators Erk and Akt

The Erk pathway plays an important role in cell differentiation, proliferation and apoptosis [20, 21], and also has a stimulating effect on BPH development [22]. To examine the effects of metformin on the downstream signaling pathway of IGF-1 in prostate epithelial cell growth, we next evaluated the protein levels of pho-Erk and pho-Akt in metformin-treated BPH-1 cells. We observed the decreased phosphorylation of Erk protein, in the wake of increased doses of metformin (Fig 4A). The administration of metformin (5 mM) for 48 hours to BPH-1 cells induced 4-fold decrease of pho-Erk expression (Fig 4C). We next determined the level of Akt, another key regulator for cell cycle, cellular proliferation and apoptosis. As expected, we found a significant decrease of pho-Akt protein level upon the treatment of metformin (Fig 4B and 4D). This observation is in line with other studies which have shown that IGF-1 is a key activator of Akt [23, 24]. Overall, our data suggests that metformin inhibits the prostate epithelial cell growth at least partly through the Erk and Akt signaling pathway.

**Fig 4:** Metformin inhibits the expression of cell proliferating regulators, Erk and Akt. A-B: Representative immunoblot of three different experiments of pho-Erk (A) and pho-Akt protein levels (B) in BPH-1 cells 48h after treatment of metformin. C-D: Quantification of the immunoblot protein levels of pho-Erk (C) and pho-Akt (D) in BPH-1 cells treated with 5 mM metformin for 48 hours by normalization to GAPDH and Akt, respectively. *, *P*<0.05, compared with control group. CTR: control, Met: metformin.

### Metformin regulates the cell cycle and the expression of cyclin D

Following our findings that metformin affects on the expression of pho-Akt and pho-Erk, we further investigated if cyclin D1, D2 and D3, proteins active in controlling the cell cycle and in initiating DNA synthesis, are modulated. We found that in BPH-1 cells, the main targets for both Akt and Erk pathways in the process of cell cycle [10, 25, 26] were significantly reduced by treatment with metformin, especially at high concentrations of 5 and 10 mM (Fig 5A). More importantly, metformin blocked the upregulation of cyclin D1, D2 and D3 induced by IGF-1 (Fig 5B). We then assumed that metformin affects the cell cycle regulations in prostatic epithelial cells. To explore this hypothesis, the populations of BPH-1 and P69 cells in different stages were analyzed by flow cytometry after administration of metformin. We found that IGF-1 led to significant reduction of cells in the phase of G_0_/G_1_ and increasing of cells in the S and G_2_/M phases both in BPH-1 (Fig 5C and 5E) and P69 cells (Fig 5D and 5F). Concomitant administration of metformin blocked the cells in the phase of G_0_/G_1_ in the presence of metformin. Simultaneously, the G_2_/M cell population was decreased from 30.48% to 18.07% in P69 cells (Fig 5D) and from 21.52% to 16.20% in BPH-1 cells (Fig 5C). These results indicate that metformin prevents the mitotic effects of IGF-1 in prostatic epithelial cells.

The article "Metformin inhibits the proliferation of benign prostatic epithelial cells" was retracted in 2024. Reasons: errors in the data; errors in the methods; errors in the images; errors in the text.

**Fig 5:** Metformin regulates cell cycle and the expression of proteins regulating cell cycle. A: Representative immunoblot analysis of cyclin D1, D2 and D3 in BPH-1 cells 48 hours after treatment of indicated dose of metformin. GAPDH was used as a loading control. B: The effect of 48-hour treatment of 100 ng/mL IGF-1 and 5 mM metformin on the expression of cyclin D1, D2 and D3 in BPH-1 cells. C-D: Flow cytometry analysis of proliferating BPH-1 (C) and P69 (D) cells 48 hours after the addition of 100 ng/mL IGF-1, 5 mM metformin or both. E-F: The population of G0/G1 cells in BPH-1 (E) and P69 (F) cells (n = 3). *, *P*<0.05 compared with the control group; #, *P*<0.05 compared with the IGF-1 treated group. CTR: non-treated control, Met: metformin.

### Metformin interrupts the effect of stromal cells on epithelial cells

Stromal-epithelial interactions play a critical role in the development of BPH, and also in this interplay we have seen that IGF-1 acts as a paracrine factor [10, 27, 28]. Therefore, we sought to determine if metformin regulates this interaction. We found that addition of murine fibroblast 3T3 CM significantly enhanced the proliferation of BPH-1(Fig 6A) and P69 cells (Fig 6B). Meanwhile, concomitant metformin-treated CM resulted in similar cell viability to that of control cells, which were treated with normal control medium (Fig 6A and 6B), indicating that metformin inhibited the proliferation of epithelial cells induced by fibroblast CM. Furthermore, in 3T3 cells, the secretion of IGF-1 was robustly inhibited by metformin from 574.31pg/ml to 197.61pg/ml (Fig 6C). Finally, we verified the above finding in human prostatic fibroblast cells. Both IGF-1R and pho-IGF-1R in BPH-1 cells were upregulated when treated with CM of human prostatic fibroblasts. This change was suppressed by metformin-treated CM (Fig 6D). Metformin treatment also inhibited the secretion of IGF-1 in human prostatic fibroblasts (Fig 6F), and inhibited the viability of BPH-1 cells (Fig 6E). Together, we propose that metformin down-regulates the effect of stromal cells on the proliferation of epithelial cells, at least partially, via inhibition of the IGF axis.

The article "Metformin inhibits the proliferation of benign prostatic epithelial cells" was retracted in 2024. Reasons: errors in the data; errors in the methods; errors in the images; errors in the text.

**Fig 6:** Metformin interrupts the effect of stromal cells on epithelial cells. A-B: The cell viability of BPH-1 (A) and P69 (B) was markedly enhanced with conditioned medium of 3T3 fibroblast cells, and was abrogated by 5 mM metformin. C: Metformin (5 mM, 24 h) inhibited the secretion of IGF-1 in 3T3 cells. D: Immunoblots of IGF-1R and pho-IGF-1R in BPH-1 cells treated with CM of human prostatic fibroblast. E: The BPH-1 cell viability after treatment with CM of human prostatic fibroblast. F: Metformin (5 mM, 24 h) inhibited the secretion of IGF-1 in human prostatic fibroblasts. *, *P*<0.05 compared with the control (CTR) group; #, *P*<0.05 compared with CM-treated group. CTR: non-treated control, Met: metformin.

## Discussion

While there are dissenting opinions, the preponderance of the evidence supports the view that patients with insulin-resistance/type 2 diabetes are at a higher risk of developing BPH and also various diabetes-associated disorders in the pathogenesis of BPH [29]. Further, epidemiological studies demonstrate insulin-resistance as an independent risk factor for BPH development [7, 8]. Therefore, whether and how the anti-diabetic drug, metformin, affects BPH development is an important clinical issue to address. As the first-line of medication for type-2 diabetes, metformin demonstrates the best risk-benefit profile when compared with other diabetic drugs. Ours and other recent data further suggest that metformin could inhibit prostate and breast cancer cell proliferation *in vitro* [15, 30, 31] and reduce the risk of cancer [32] *in vivo*, while only moderately inhibiting benign prostatic epithelial cell growth at low concentrations (up to 5 mM) [33]. In this study, for the first time, we show that metformin potently inhibits the proliferation of human benign prostatic epithelial cells in *vitro* in a dose-dependent (0.5, 1, 5, and 10 mM) and time-dependent (6, 12, 24, and 48h) manner. Furthermore, we find that IGF-1 is involved in the abrogation of cell proliferation induced by metformin. Taken together, our data suggest that metformin reduces the proliferation of prostatic epithelial cells.

Meanwhile, it is worthy to investigate the underlying molecular mechanism of metformin regulating prostatic epithelial cell proliferation. The IGF-1 signaling pathway has been identified both in normal prostate gland development and in prostatic cancer cell progression and studies have shown that locally enforced IGF-1 expression induces hyperplasia in the prostate [19, 34]. In our previous study, we found that stromally secreted IGF-1 stimulates BPH-1 cellular proliferation via up-regulation of epithelial mitogen-activated protein kinase, Akt, and cyclin D protein levels, while simultaneous down-regulation of cyclin-dependent kinase inhibitor p27. The results suggest that the activation of the IGF-1 axis is critical in prostatic epithelial cell growth [10]. Here, we provide evidence that metformin down-regulates the IGF-1 axis through inhibiting the phosphorylation of IGF-1R in a time- and dose-dependent manner. Moreover, metformin suppressed the activation of IGF-1R stimulated by IGF-1. Collectively, our data suggest that the suppressive effect of metformin on prostatic epithelial cellular proliferation is at least partially attributed to the suppression of the IGF-1 axis.

The article "Metformin inhibits the proliferation of benign prostatic epithelial cells" was retracted in 2024. Reasons: errors in the data; errors in the methods; errors in the images; errors in the text.

Another observation in our study is that the inhibiting effect of metformin on the proliferation of benign prostatic epithelial cells mainly attributes to the regulation of cell cycle. It has been shown that the cyclin D family (cyclin D1, D2 and D3), a major regulator of core cell cycle machinery [15, 25, 35], is a main downstream target of the IGF-1 axis [10, 36–38]. We have found that BPH-1 cell proliferation was markedly enhanced with over-expression of cyclin D [10]. Therefore, the IGF-regulated cyclin expression might be a potential molecular target in order to control BPH development. As shown in Figs 4 and 5, this hypothesis is confirmed by the cell cycle blockage in the G0/G1 phase and the inhibition of cyclin protein expression with the administration of metformin.

Stromal-epithelial interactions play a pivotal role in the regulation of the development and growth of the prostate. The study of Dong et al. found a 3-fold higher expression of IGF-IR and a 10-fold higher expression of IGF-II in primary culture of BPH stromal cells when compared with normal stromal cells [39]. In line with previous reports, we have also shown that stromally secreted IGF-1 could act as a paracrine factor and directly induce the proliferation and growth of prostatic epithelial cells [10]. Furthermore, here we demonstrate that metformin decreases the secretion of IGF-1 from the stromal cells and inhibits the proliferation of prostatic epithelial cells in metformin pre-treated CM from stromal cells. These results suggest that metformin affects the stromal and epithelial cell interactions not only through inhibiting the expression of IGF-1R and the activation of the IGF-1 axis in the epithelial cells, but also through regulating the stromally secreted IGF-1. Further investigation of this pathway may be helpful in the management of lower urinary tract symptoms suffering from BPH in diabetic patients.

The article "Metformin inhibits the proliferation of benign prostatic epithelial cells" was retracted in 2024. Reasons: errors in the data; errors in the methods; errors in the images; errors in the text.

In conclusion, our study provides the first demonstration that metformin significantly inhibits the proliferation of benign prostatic epithelial cells. We show that metformin lowers the G2/M cell population and simultaneously increases the G0/G1 population. Furthermore, we demonstrate that metformin not only inhibits the cell proliferation and IGF-1R expression activated by IGF-1, but also inhibits the IGF-1 secretion in stromal cells and then suppresses the epithelial cell proliferation with stromal CM. Findings here might have significant clinical implications in management of BPH patients treated with metformin.
